The article "Effects of Competition and Facilitation on Species Assemblage in Two Types of Tropical Cloud Forest" was published in 2013. Journal: PLoS One.

# Effects of Competition and Facilitation on Species Assemblage in Two Types of Tropical Cloud Forest

**DOI:** 10.1371/journal.pone.0060252

**Published:** 2013-04-02

**Authors:** Wenxing Long, Runguo Zang, Yi Ding, Yunfeng Huang

**Affiliations:** 1 Key Laboratory of Protection and Development Utilization of Tropical Crop Germplasm Resource, Ministry of Education, College of Horticulture and Landscape Agriculture, Hainan University, Haikou, Peoples Republic of China; 2 Key Laboratory of Forest Ecology and Environment of State Forestry Administration, Institute of Forest Ecology, Environment and Protection, Chinese Academy of Forestry, Beijing, Peoples Republic of China; University of Florida, United States of America

## Abstract

Competition and facilitation between tree individuals are two kinds of non-random processes influencing the structure and functioning of forest communities, but how these two plant-plant interactions change along gradient of resources or environments remains very much a matter of debate. We developed a null model to test the size-distance regression, and assessed the effects of competition and facilitation (including interspecific interactions, intraspecific interactions and overall species interactions) on each adult tree species assemblage [diameter at breast height (dbh) ≥5 cm] across two types of tropical cloud forest with different environmental and resource regimes. The null model test revealed that 17% to 27% tree species had positive dbh-distance correlations while 11% to 19% tree species showed negative dbh-distance correlations within these two forest types, indicating that both competition and facilitation processes existed during the community assembly. The importance of competition for heterospecific species, and the intensity of competition for both heterospecific and overall species increased from high to low resources for all the shared species spanning the two forests. The importance of facilitation for conspecific and overall species, as well as that the intensity of facilitation for both heterospecific and conspecific species increased with increasing low air temperature stress for all the shared species spanning the two forests. Our results show that both competition and facilitation processes simultaneously affect parts of species assemblage in the tropical cloud forests. Moreover, the fact that nearly 50% species assemblage is not detected with our approaches suggest that tree species in these tropical forest systems are assembled with multiple ecological processes, and that there is a need to explore the processes other than the two biotic interactions in further researches.

## Introduction

Negative and positive interactions between tree individuals are two kinds of non-random processes, frequently regarded as having central roles in influencing the structure and functioning of forest communities [1], [2], [3], [4], [5], [6]. For example, competition is the tendency of neighboring plants to utilize the same resources such as light, soil nutrients, water, or space [1]; while facilitation, which is the most common example of positive plant-plant interaction, refers to that fitness of one plant species benefits from the improved (micro) environmental conditions created directly or indirectly by neighboring plants, and outweighs the costs of living close to other individual [3].

Intensity and importance are defined as the two distinct parameters necessary for understanding the role of competition in forest species assembly [4], [7], [8], [9]. The intensity of competition is its absolute impact, and the importance of competition is its impact relative to that of all the factors in the environment that influence plant success [7], [10]. Changes in competition intensity with resources and environmental conditions remain very much a matter of debate [4], [9], with those involved roughly grouped into two opposing dominant groups. One group postulates that competition remains equivalent across resource gradients [2], [11], [12], whereas the other group argues that competition changes across resource gradients [1]. Some studies suggest that competition intensity increases as resource availability becomes richer [10]. Commonly cited examples are the prediction that maximum species height is higher and that the role of competition increases in more productive environments [13]. Opposing examples to this have been observed in plant communities in which competition intensity remains unchanged [14], [15], or declines with available resources [16]. Coexisting species can differ in their response to maintain performance under neighbor competition and in their stress tolerance [15].

Species in stressful environmental conditions usually exhibit facilitation due to amelioration by neighbors favoring growth over competition for resources with the same neighbors, which impair growth [3]. This positive interaction plays great roles in species generation [17], species distribution [6], community diversity [18], community structure and dynamics [19], [20]. For example, Maetre et al. found that lichens in a semi-arid Mediterranean environment coexist through facilitation, which is dependent on the type of abiotic stress and the spatial scale considered [5]. These beneficial impacts of neighbors usually increase with increasing severity, and have been proven in study systems such as low temperature alpine forests [3], arid shrub communities [18], and so on.

A common method for exploring the influence of plant-plant interactions along gradients of resources or environments in mature, natural communities is the size-distance regression approach as advocated by Welden and Slauson [7]. For example, the size-distance regression assumes that competitive interference between neighboring plants, if present, will manifest through a reduction in the size of one or both competing neighbors [21], [22], [23]. However, a lack of null model test makes this approach not easily distinguish competition from other processes (e.g. facilitation process), and thus obscures the effect of both competition and facilitation on species assemblage. This null model approach has been tailored to distinguish both the negative and positive interactions from the stochastic process influencing community assembly [24]. An incorporation of null model tests into size-distance regression approach thus can provide an opportunity to distinguish both the competition and facilitation from stochastic process.

Tropical cloud forest is mainly found in tropical parts of the Americas, Africa and Asia [25]. Trees in cloud forests are typically more malformed (i.e. twisted and misshapen) and elfin, and covered in more epiphytes. Environmental conditions in these forests are characterized by low air temperature, strong winds, frequent fog, and high levels of ultraviolet radiation compared with lower altitude forests [26], [27], [28]. Plants in these forests often tolerate with environmental stresses such as low total nitrogen, low total phosphorus and low air temperature [28], [29], [30].

In this study, we developed a null model, and expected that integration of this null model test with size-distance regression can help distinguish competition from facilitation. Then we explored patterns of absolute impacts and relative impacts for competition and facilitation on each adult tree species assemblage [diameter at breast height (dbh) ≥5 cm], between two tropical cloud forests with different degree of environmental stresses and forest resources. We hypothesized that (1) an incorporation of null model test into size-distance analysis would help distinguish competition process from facilitation process; and (2) both the importance and intensity of competition and facilitation would increase with decreasing forest resources and increasing low temperature stress in the two types of tropical cloud forest.

## Materials and Methods

### Study Sites

This study was conducted in a tropical montane evergreen forest (TMEF) and a tropical dwarf forest (TDF) in the Bawangling Nature Reserve (BNR) (18°50′ –19°05′ N, 109°05′ –109°25′ E), Hainan Island, South China (Figure 1). The location of our study was permitted by the Administration Bureau of BNR. BNR is *ca.* 500 km^2^ in area, with an altitude range of *ca.* 100–1654 m a.s.l. The mean annual temperature is 23.6°C, and annual precipitation is 1677.1 mm at *ca.* 100 m altitude, with a distinct wet season from May to October and a dry season from November to April [31]. The TDF (19°05′04.8″ N, 109°12′43.5″ E) is mainly distributed around the mountain tops at altitudes over 1250 m (Figure 1), and has montane meadow soils developed from sandstone. with the mean daily air temperature from May to October ranging from 17.72±0.82°C to 20.43±1.29°C and photosynthetic photon flux density (PPFD) in June ranging from 17.01±8.82 µmol m^−2^ s^−1^ to 48.45±12.30 µmol m^−2^ s^−1^; while the TMEF (19°05′24.5″ N, 109°12′56.2″ E) is adjacent to TDF (Figure 1), mainly distributed at an altitude between 1200 m –1300 m, and has montane yellow soils developed from granite, with the mean daily air temperature from May to October ranging from 19.22±2.81°C to 25.04±0.22°C and PPFD in June ranging from 7.15±1.27 µmol m^−2^ s^−1^ to 19.65±2.41 µmol m^−2^ s^−1^ [28], [32]. These two types of forest are primary old-growth forests, and usually collectively classified as tropical cloud forest due to the high altitude of their occurrence and frequent covering of fog.

**Figure 1:** The location of the study plots. Our study forests, including tropical montane evergreen forests (TMEF) and tropical dwarf forests (TDF), located in the Bawangling Nature Reserve (BNR) in Hainan Island, South China.

Compared with TMEF, TDF is an unproductive forest community with lower total nitrogen, lower total phosphorus and lower organic matter [28]. The mean daily air temperature from May to Oct. is 21.76±2.44°C and 19.33±1.03°C in TMEF and TDF, respectively [28]. This low air temperature stress has been proven to be an environmental filter constraining tropical cloud forest species composition and distribution [29], [30].

### Data Collection

Four 50×50 m plots were located within the TMEF and TDF sites (each with four plots), respectively, using a random number table to determine location. Our dataset is confined to such plot size because forest in TDF is often discontinuously distributed around the mountain tops, this size thus is maximal in TDF which can be comparable with that in TMEF. The study plots in TMEF and TDF were located on an eastern slope with the inclination ranging from 30° to 45°, with the altitude in TMEF ranging from 1220 m to 1270 m and that in TDF ranging from 1260 m to 1340 m. Each plot was subdivided into twenty five 10×10 m subplots using an electronic total station (Leica TSP1200+; Heerbrugg, Switzerland), and each 10×10 m subplot was subdivided into four 5×5 m quadrates for precisely measuring the tree coordinates. All free standing trees with diameter at breast height (dbh, 1.3 m above the ground) ≥5 cm were mapped (Figure 2) and identified to species in accordance with Flora Reipublicae Popularis Sinicae [33]. The geographic coordinates of all the free standing trees were recorded following a standard field protocol [34]. Species with more than six individuals were chosen to assess size-distance regression to avoid the “dilution effects” [24].

**Figure 2:** The spatial distribution of individual trees in each forest type. The diameter at breast height (dbh) of each tree was over 5 cm. The sizes of individual circles were represented by the dbh of individual trees. There were four plots in tropical dwarf forests (TDF1, TDF2, TDF3 and TDF4) and tropical evergreen forests (TMEF1, TMEF2, TMEF3 and TMEF4), respectively.

### Data Analysis

We assessed the size-distance regression for each species in each plot. Size referred to the sum of the dbh of the four nearest neighbors plus the dbh of the focal tree. Distance referred to the sum of the distance of the four nearest neighbors to that focal tree [22]. The coefficient of determination r^2^ was taken as the estimate of the importance of competition or facilitation, and the slope of regression was taken as the estimate of the intensity of competition or facilitation [7]. “Nearest neighbors” referred to the four nearest neighbors of a focal tree. Trees with a “conspecific neighborhood” had three or four conspecific nearest neighbors, and trees with a “heterospecific neighborhood” had none or one conspecific nearest neighbor. The dbh-distance regression was conducted for inferring overall species, intraspecific, and interspecific competition by respectively including only one of the following subsets of focal trees in the analysis: all focal trees of a given species, focal trees with a conspecific neighborhood, and focal trees with a heterospecific neighborhood.

We established a null model to show that dbh and nearest neighbor distance were not correlated for each tree species, implying that stochastic processes affect species assemblage. We fixed the observed richness and abundances for each species, as well as the geographic coordinates for each individual tree in a 2500 m^2^ plot, but assigned dbh values extracted from all individuals in the plots to individual trees randomly without replacement. Next, we tested the regression between dbh and nearest neighbor distance for each tree species, and calculated the expected coefficient of determination r^2^. For each tree species, we generated distribution of the expected coefficient of determination r^2^ with 9999 random permutations of the dbh matrix. If the observed coefficient of determination r^2^ fell within the 5th and 95th percentiles of the expected r^2^, the null hypothesis could not be rejected; otherwise, we would conclude that a significant correlation was presented between dbh and nearest neighbor distance for the tree species, and would infer that the species were assembled with a non-random process (i.e. a negative interaction or a positive interaction).

The non-random processes inferring from significant dbh-distance regressions were grouped into negative interactions and positive interactions (Figure 3). According to the slope for size-distance regressions, first, in case the slope >0, a significant positive correlation between dbh and nearest neighbor distance indicates an inhibition in growth or size of a plant by another, and this negative interaction can also be termed as competition. Thus, r^2^ and slope were taken as the importance and intensity of competition, respectively. Second, in case the slope <0, a significant negative correlation between dbh and nearest neighbor distance indicates amelioration in growth or size of a plant by another, and this positive interaction can be termed as facilitation. r^2^ and slope, therefore, were taken as the importance and intensity of facilitation, respectively.

**Figure 3:** A predictive framework indicating significant positive and negative size-distance correlations for tree species. The two categories of correlations were assumed to differ significantly from those that individual trees were distributed stochastically, and the size and nearest neighbor distance therefore were not correlated. Significant positive correlation between size and nearest neighbor distance would predict a negative interaction (i.e. competition process) on species assemblage (A), and significant negative correlation between size and nearest neighbor distance would predict a positive interaction (i.e. facilitation process) on species assemblage (B).

Differences in average tree density and average dbh between TMEF and TDF were assessed with Wilcoxcon test. For the shared species spanning TMEF and TDF, differences in intensity and importance of interspecific interactions, intraspecific interactions, and overall species interactions for both competition and facilitation between these two types of forest, were assessed using a paired student’s test. When there were no significant differences for the above parameters between TMEF and TDF, a linear mixed model (lme function) was used to analyze the variance explained by the forest type which was regarded as random variable in the tests, as well as species variable. All statistical analyses were performed with the R 2.9.2 program [35].

## Results

### Stand Structure Across the Two Types of Tropical Cloud Forest

There were 73 and 66 tree species with dbh ≥5 cm in TMEF and TDF, respectively. The common dominant families were Lauraceae, Symplocaceae, Rubiaceae, Fagaceae and Oleaceae. The common dominant genera were *Symplocos*, *Syzygium*, *Cyclobalanopsis*, *Lithocarpus* and *Beilschmiedia*. The tree density differed non-significantly between TMEF and TDF (Wilcoxcon test, *W* = 14, *P* = 0.11; TMEF: 576.8±38.0 stems per 2500 m^2^, TDF: 694.3±108.6 stems per 2500 m^2^), while the average dbh differed significantly between these two forest types (Wilcoxcon test, *W* = 16, *P* = 0.03; TMEF: 12.0±0.2 cm, TDF: 10.2±0.1 cm). There were 18 common species spanning both TMEF and TDF with a great abundance (Table 1).

**Table 1:** Average abundance and diameter at breast height (dbh) of live trees ≥5.0 cm (mean ± SD) in 2500 m^2^ plots, for the shared species spanning tropical montane evergreen forest (TMEF) and tropical dwarf forest (TDF).

Species	TMEF			TDF		
	Abundance	Maximum dbh	Mean dbh	Abundance	Maximum dbh	Mean dbh
*Syzygium araiocladum*	88.5±49.9	14.7±2.8	7.6±0.5	23.3±13.8	15.0±1.1	9.1±0.9
*Syzygium buxifolium*	74.3±11.6	31.3±9.9	11.1±1.5	96.3±24.1	25.8±5.9	10.0±1.3
*Distylium racemosum*	59.8±18.8	34.1±5.0	15.8±0.7	147.8±105.4	32.4±9.4	12.6±0.8
*Cyclobalanopsis disciformis*	59.5±17.9	38.2±5.3	18.1±2.0	23.3±15.0	31.7±7.6	13.3±2.2
*Ternstroemia gymnanthera*	52.0±11.7	29.9±8.3	11.9±1.7	14.5±2.4	26.0±5.2	10.7±0.5
*Dacrydium pierrei*	24.3±6.9	47.9±17.1	21.0±4.0	21.2±3.4	40.8±2.0	19.18±1.1
*Pentaphylax euryoides*	21.8±4.1	25.0±4.7	10.6±1.8	17.0±15.6	18.2±3.4	10.0±0.5
*Symplocos lancifolia*	19.3±8.8	15.7±3.5	9.4±1.7	23.3±14.8	14.8±8.1	7.2±1.7
*Rhododendron moulmainense*	17.8±3.3	12.9±4.1	7.9±1.2	18.3±5.7	12.6±0.8	7.5±0.4
*Engelhardtia roxburghiana*	16.8±1.9	24.6±5.6	11.4±0.8	50.3±24.5	22.2±4.4	8.6±1.0
*Gordonia axillaris*	16.5±0.7	12.5±1.4	7.6±0.5	20.3±9.5	25.8±11.6	9.2±1.6
*Symplocos poilanei*	11.0±4.6	8.7±0.8	6.4±0.4	26.3±17.7	11.7±4.0	6.6±0.3
*Rapanea neriifolia*	11.0±6.2	14.4±1.5	9.2±1.2	14.3±6.9	14.8±2.5	9.7±1.5
*Exbucklandia tonkinensis*	10.7±3.5	39.8±12.6	16.7±4.3	11.0±7.1	27.5±7.2	16.2±3.5
*Osmanthus didymopetalus*	8.8±2.2	15.1±4.9	9.7±1.7	14.5±3.4	16.0±6.4	8.6±0.1
*Michelia mediocris*	8.0±2.2	23.4±8.2	14.7±1.6	14.7±10.3	26.6±10.1	12.5±3.1
*Acronychia pedunculata*	7.7±1.2	13.8±1.9	8.6±0.7	17.0±13.5	16.5±4.1	8.3±0.4
*Cyclobalanopsis championii*	7.0±0	40.3±3.3	27.6±0.5	9.5±4.9	59.8±25.8	26.1±0.6

### Percentage of Tree Species in Competition and Facilitation Across the Two Types of Tropical Cloud Forest

There were 41±4% and 37±2% heterospecific species (Figure 4A), 43±4% and 38±7% conspecific species (Figure 4B), and 28±2% and 44±5% overall species (Figure 4C) in TMEF and TDF, respectively, showed significant correlations between dbh and nearest neighbor distance using null model tests, indicating that non-random processes (i.e. competition or facilitation) influence species assemblage in the two types of tropical cloud forest.

**Figure 4:** Percentage of heterospecific species, conspecific species and overall species showing significant positive and negative dbh-distance correlations. The three types of dbh-distance correlations showing the non-random, competition and facilitation processes affecting on tree species assemblage, respectively.

There were 23±3% and 26±5% heterospecific species (Figure 4A), 27±5% and 19±9% conspecific species (Figure 4B), and 17±8% and 27±7% overall species (Figure 4C) in TMEF and TDF, respectively, showed significant positive correlations between dbh and nearest neighbor distance using null model tests. These figures indicate that interspecific competition, intraspecific competition, and overall species competition influence species assemblage.

With respect to significant negative correlations between dbh and nearest neighbor distance, there were 11±4% and 18±5% heterospecific species (Figure 4A), 19±3% and 18±5% conspecific species (Figure 4B), and 17±7% and 11±4% overall species (Figure 4C) in TMEF and TDF, respectively. These figures indicate that interspecific facilitation, intraspecific facilitation, and overall species facilitation influence species assemblage in the two types of tropical cloud forest.

### Patterns of Importance and Intensity of Competition Across the Two Types of Tropical Cloud Forest

The coefficient of determination r^2^ for positive dbh-distance regression, which was interpreted as the percentage variance of dbh explained by nearest neighbor distance, was taken as the estimate of importance of competition. For the shared species spanning TMEF and TDF and assembled with competition processes, paired *t*-tests revealed that the importance of interspecific competition was significantly higher in TDF than TMEF (*t* = −2.32, df = 15.32, *P* = 0.03; Table 2), while the importance of intraspecific competition and importance of overall species competition differed non-significantly between these two forest types (intraspecific competition: *t* = −0.16, df = 15.78, *P* = 0.87; overall species competition: *t* = −1.08, df = 9.96, *P* = 0.30). A linear mixed model showed that forest type accounted for 0.06% and 1.51% of the variance for the importance of intraspecific competition and overall species competition, respectively.

**Table 2:** Comparison in importance (coefficient of determination for positive dbh-distance regression) of interspecific competition (heterospecific neighbors), intraspecific competition (conspecific neighbors) and overall species competition (all neighbors) between tropical montane evergreen forest (TMEF) and tropical dwarf forest (TDF) for the shared species occupying these two forests.

Heterospecific neighbors			Conspecific neighbors			All neighbors		
Species	TMEF	TDF	Species	TMEF	TDF	Species	TMEF	TDF
*Michelia mediocris*	0.680	0.551	*M. mediocris*	0.738	0.240	*Exbucklandia tonkinensis*	0.415	0.388
*Gordonia axillaris*	0.002	0.149	*E. tonkinensis*	0.682	0.004	*Engelhardtia roxburghiana*	0.411	0.127
*Cyclobalanopsis disciformis*	0.063	0.699	*C. disciformis*	0.268	0.338	*Dacrydium pierrei*	0.198	0.140
*Symplocos lancifolia*	0.256	0.461	*S. lancifolia*	0.354	0.769	*Rhododendron moulmainense*	0.150	0.274
*C. championii*	0.00005	0.648	*E. roxburghiana*	0.245	0.540	*Rapanea neriifolia*	0.0002	0.931
*D. pierrei*	0.123	0.722	*R. moulmainense*	0.001	0.1964	*Syzygium buxifolium*	0.077	0.141
*R. moulmainense*	0.004	0.122	*Osmanthus didymopetalus*	0.00003	0.003	*S. araiocladum*	0.0003	0.216
*Distylium racemosum*	0.080	0.015	*D. racemosum*	0.054	0.285			
*S. araiocladum*	0.116	0.350	*Pentaphylax euryoides*	0.173	0.317			

Note: The r square of each species is calculated from the mean of all plots in that forest type.

The slope of the positive dbh-distance regression was taken as the estimate of the competition intensity. Paired *t*-tests showed that the intensity of interspecific competition was significantly higher in TDF than TMEF (*t* = −3.24, df = 8, *P* = 0.01; Table 3), and that the intensity of overall species competition as well was marginally significantly higher in TDF than TMEF (*t* = −2.12, df = 6.42, *P* = 0.07). However, the intensity of intraspecific competition exhibited no significant difference between the two forest types (*t* = −1.67, df = 12.22, *P* = 0.12), with the forest type accounting for 0.003% of the variance using a linear mixed model.

**Table 3:** Comparison in intensity (slope for positive dbh-distance regression) of interspecific competition (heterospecific neighbors), intraspecific competition (conspecific neighbors) and overall species competition (all neighbors) between tropical montane evergreen forest (TMEF) and tropical dwarf forest (TDF), for the shared species occupying these two forests.

Heterospecific neighbors			Conspecific neighbors			All neighbors		
Species	TMEF	TDF	Species	TMEF	TDF	Species	TMEF	TDF
*Michelia mediocris*	0.037	0.119	*M. mediocris*	0.525	0.690	*Exbucklandia tonkinensis*	0.076	0.208
*Gordonia axillaris*	0.006	0.048	*E. tonkinensis*	0.114	1.493	*Engelhardtia roxburghiana*	0.062	0.063
*Cyclobalanopsis disciformis*	0.033	0.061	*C. disciformis*	0.080	0.277	*Dacrydium pierrei*	0.041	0.057
*Symplocos lancifolia*	0.066	0.185	*S. lancifolia*	0.692	0.767	*Rhododendron moulmainense*	0.034	0.051
*C. championii*	0.001	0.066	*E. roxburghiana*	0.211	0.278	*Rapanea neriifolia*	0.003	0.455
*D. pierrei*	0.054	0.088	*R. moulmainense*	0.035	0.468	*Syzygium buxifolium*	0.030	0.063
*R. moulmainense*	0.004	0.028	*Osmanthus didymopetalus*	0.032	0.103	*S. araiocladum*	0.002	0.198
*Distylium racemosum*	0.037	0.045	*D. racemosum*	0.043	0.109			
*S. araiocladum*	0.001	0.003	*Pentaphylax euryoides*	0.188	0.250			

Note: The slope of each species is calculated from the mean of all plots in that forest type.

### Patterns of Importance and Intensity of Facilitation Across the Two Types of Tropical Cloud Forest

For the shared species spanning TMEF and TDF and assembled with facilitative processes, the importance of intraspecific facilitation and overall species facilitation was significantly higher in TDF than TMEF (Intraspecies facilitation, *t* = −2.67, df = 19.87, *P* = 0.01; Overall species facilitation, *t* = −3.24, df = 12.95, *P = *0.006; Table 4); while the importance of interspecific facilitation differed non-significantly between these two forest types (*t* = −1.696, df = 13.23, *P* = 0.12), in which the forest type only accounted for 5.92% of the variance using a linear mixed model.

**Table 4:** Comparison in importance (coefficient of determination for negative dbh-distance regression) of interspecific facilitation (heterospecific neighbors), intraspecific facilitation (conspecific neighbors) and overall species facilitation (all neighbors) between tropical montane evergreen forest (TMEF) and tropical dwarf forest (TDF), for the shared species occupying these two forests.

Conspecific neighbors			Heterospecific neighbors			All neighbors		
Species	TMEF	TDF	Species	TMEF	TDF	Species	TMEF	TDF
*Cinnamomum tsoi*	0.430	0.640	*Acronychia pedunculata*	0.376	0.586	*Cryptocarya chinensis*	0.009	0.516
*Cyclobalanopsis disciformis*	0.0000007	0.00003	*C. chinensis*	0.00002	0.536	*C. disciformis*	0.001	0.199
*Distylium racemosum*	0.010	0.230	*D. racemosum*	0.0001	0.00009	*Ficus variolosa*	0.196	0.570
*Ervatamia officinalis*	0.080	0.630	*Elaeocarpus howii*	0.00005	0.958	*Lyonia rubrovenia*	0.188	0.721
*Illicium ternstroemioides*	0.100	0.550	*F. variolosa*	0.352	0.561	*Podocarpus neriifolius*	0.423	0.472
*Machilus velutina*	0.010	0.390	*Osmanthus didymopetalus*	0.602	0.179	*Rhododendron moulmainense*	0.000001	0.166
*Pentaphylax euryoides*	0.520	0.590	*Podocarpus neriifolius*	0.351	0.954	*Symplocos poilanei*	0.181	0.392
*Rapanea neriifolia*	0.290	0.920	*S. lancifolia*	0.001	0.0002	*Ternstroemia gymnanthera*	0.126	0.282
*R. moulmainense*	0.220	0.710	*Syzygium araiocladum*	0.157	0.236			
*S. poilanei*	0.620	0.920						
*Xanthophyllum hainanense*	0.670	0.680						

Note: The r square of each species is calculated from the mean of all plots in that forest type.

The intensity of interspecific facilitation was significantly higher in TDF than TMEF (*t* = −2.588, df = 14.53, *P = *0.021; Table 5), as well as that the intensity of intraspecific facilitation was marginally significantly higher in TDF than TMEF (*t* = −2.118, df = 15.88, *P = *0.050). However, the intensity of overall species facilitation exhibited no significant difference between the two forest types (*t* = −1.273, df = 18.63, *P = *0.219), in which the forest type only accounted for 4.71% of the variance.

**Table 5:** Comparison in intensity (slope for positive dbh-distance regression) of interspecific facilitation (heterospecific neighbors), intraspecific facilitation (conspecific neighbors) and overall species facilitation (all neighbors) between tropical montane evergreen forest (TMEF) and tropical dwarf forest (TDF), for the shared species occupying these two forests.

Conspecific neighbors			Heterospecific neighbors			All neighbors		
Species	TMEF	TDF	Species	TMEF	TDF	Species	TMEF	TDF
*Cinnamomum tsoi*	0.311	0.736	*Acronychia pedunculata*	0.096	0.090	*Cryptocarya chinensis*	0.009	0.095
*Cyclobalanopsis disciformis*	0.0001	0.001	*Cryptocarya chinensis*	0.0003	0.098	*C. disciformis*	0.003	0.036
*Distylium racemosum*	0.017	0.182	*D. racemosum*	0.0005	0.002	*Ficus variolosa*	0.087	0.132
*Ervatamia officinalis*	1.189	3.150	*Elaeocarpus howii*	0.001	0.132	*Lyonia rubrovenia*	0.070	0.348
*Illicium ternstroemioides*	0.181	0.393	*F. variolosa*	0.079	0.075	*Podocarpus neriifolius*	0.267	0.100
*Machilus velutina*	0.041	0.429	*Osmanthus didymopetalus*	0.072	0.178	*Rhododendron moulmainense*	0.0003	0.070
*Pentaphylax euryoides*	0.377	1.149	*Podocarpus neriifolius*	0.003	0.221	*Symplocos poilanei*	0.044	0.078
*Rapanea neriifolia*	0.214	1.048	*S. lancifolia*	0.002	0.061	*Ternstroemia gymnanthera*	0.053	0.117
*R. moulmainense*	0.298	3.951	*Syzygium araiocladum*	0.024	0.061			
*S. poilanei*	0.756	1.543						
*Xanthophyllum hainanense*	1.522	1.888						

Note: The slope of each species is calculated from the mean of all plots in that forest type.

## Discussion

### Null Model Test and dbh-distance Analysis

As expected, the null model test approach, which hypothesized that plant dbh did not correlate with the nearest neighbor distance, and that the stochastic processes affected species assemblage [24], helps us recognize both the positive and negative dbh-distance correlations for tree species in TMEF and TDF (Figure 4; Table 2, 4). Thus, our study demonstrates that both competition and facilitation processes affect the species assemblage of the tropical cloud forest communities. The integration of the null model test into the dbh-distance regression analysis, therefore, can help us distinguish competition process from facilitation process, allowing the accurate assessment of the effect of these two processes on community structuring. Our approaches may be complementary to the research of Shackleton and Getzin *et al*. [22], [23], in which the competition process was obscured with other processes (e.g. the facilitation process) due to the lack of null model tests, and the effect of competition was probably overestimated. Furthermore, our approaches have the advantage of assessing the influence of competition and facilitation on species assemblage at the community level, and thus might be superior to short-time manipulative experiments which only focus on one or part of species assemblage in communities [36].

Although both competition and facilitation influence species coexistence in tropical cloud forests, our results reveal that the roles of these two processes are relatively small, with the average percentage of species assembled by these two interactions both less than 30 (e.g. competition: 17% to 27% species; facilitation: 11% to 19% species). The relatively low percentage of species organized by competition process is a possible result of the niche differentiation stabilizing the coexistence of species with dbh over 5 cm; interactions among these species are weak probably due to high mortality from seedings to adult trees [37]. Facilitation can be caused by microhabitat heterogeneity, such as the variability in forest-floor micro-relief [18], light [38], and soil properties [39]), which consequently lead to species aggregation distribution for one hand [40]. In this study, the location of tropical cloud forests at high altitudes may expose species to the disadvantages of low air temperature stress [29], [30]. Some adult tree species in this stressful condition probably only serve as nurse plants instead of amelioration by neighbors [3], leading to small proportion of species assembled by facilitation. Additionally, some ecological processes such as stochastic demographic processes [41], disturbances [42], and environmental heterogeneity [29], [30], [43], may also affect species assemblage in tropical forests [43]. For example, the strong winds in the tropical cloud forests is an important disturbance [26], [27], [28], and may impose filtering on species coexistence [44]; in TDF, the low air temperature has been proven to be an environmental filtering on species assemblage by affecting functional trait variation [30]. The rest nearly 50% of species, therefore, can be assembled by these ecological processes. Alternatively, our study suggests that there are multiple processes affecting species assemblage in these two tropical forest systems.

### Patterns of Importance and Intensity of Competition

The coefficient of determination r^2^ for the positive dbh-distance regression, taken here as an estimate of the importance of competition [7], varied a great deal in the tropical cloud forests (Table 2), indicating a variation in the importance of competition for the different tree species assemblage. In our study, species affected by competition process mainly belong to Fagaceae, Myrtaceae, Magnoliaceae and Hamamelidaceae (Table 2). However, for the species affected by competition effects, the importance of interspecific competition, intraspecific competition, and overall species competition was all lower than 0.50, suggesting that ecological processes other than competition, such as disturbance, herbivores, plant diseases, and facilitation effect, typically act to determine these species assemblage in the forest communities [43], [45]. The importance of both interspecific competition and overall species competition for the shared species spanning TMEF and TDF was lower in TMEF than TDF (Table 2), contrasting with our expectations. This finding suggests that species in TMEF are more sensitive to other biotic and abiotic factors than TDF. As such, soil nutrients and light are more heterogeneous in TMEF [29], and disturbances increase in TMEF due to lower altitudinal forest distribution compared with TDF; thus, the relative impacts of other biotic factors and abiotic factors are more pronounced in TMEF than TDF.

Contrary to the hypothesis, the intensity of both interspecific competition and overall species competition for the shared species spanning TMEF and TDF are statistically lower in a productive forest (i.e. TMEF) than in an unproductive forest (i.e. TDF) (Table 3), indicating that competition intensity increases with decreasing forest resources. Our result contrasts with the theoretical predictions by Tilman and Grime [1], [2], [11], [12], in which competition intensity across resource gradients either remains unchanged, or is high in productive sites. Moreover, our result is also inconsistent with the manipulative experiments by DiTomasso and Aarssen [14], in which the general intensity of competition neither increases nor decreases with increasing nutrient levels. But our result agrees with the research conducted by Goldberg *et al*. in plant communities and by Dhondt in bird communities [16], [46]. Alternatively, all of these studies may prove that intensity of competition does not vary consistently with resource levels [47]. Patterns of competition intensity in the present study may be related to the soil nutrients; for example, differences in the soil phosphorus between TMEF and TDF. Phosphorus has been recognized as a limiting factor in tropical forests [48], and has been demonstrated to influence plant growth and species distribution in the studied tropical cloud forests [29]. Species may compete more intensively for limiting soil phosphorus in TDF than TMEF because soil phosphorus limitation is more significant in TDF than TMEF [28]. A further explanation can be linked to the differences in below-ground competition intensity; above- and belowground competition usually exhibit positive interactions [49]. For example, compared with TDF, higher soil depth in TMEF may allow the plant fine roots to be more widely distributed at different soil profiles; species in TMEF can partition below-ground resources more efficiently and thus can avoid direct competition [50].

### Patterns of Importance and Intensity of Facilitation

The importance of intraspecific facilitation and overall species facilitation was significantly higher in TDF than TMEF (Table 4), suggesting that facilitation process plays a more important role in species assemblage in TDF than TMEF. Our results thus demonstrate the evidence that species composition and distribution in high altitude (i.e. subalpine or alpine) forest communities are easy to be facilitated by neighboring organisms [3], [18]. In our study, the species influenced by facilitation process mainly belong to Lauraceae, Ericaceae and Symplocaceae (Table 4). Species in tropical cloud forests can tolerate low air temperature constraint, which lead to the slow growth and relative small final plant sizes [29], [30]. The amelioration of this severe low air temperature stress by neighbors may favor growth more than competition for resources with the same neighbors, which impair growth [3]. For example, melioration by some neighboring plant species and individuals probably makes the temperature environment inside the communities higher and more stable than that outside the communities during the growing periods [51], which is helpful to the plant species growth. The increasing facilitative intensity from TMEF to TDF may result from the increasing low air temperature stress (Table 5). Thus our studies lend a support the stress gradient hypothesis [3], [5], [18].

### Conclusions

Our approaches of combining null model tests with dbh-distance regression approaches make it possible to detect the effects of competition and facilitation on species assemblage in tropical cloud forests. The importance of competition and the competition intensity for the shared species spanning the two forest types increase with decreasing forest resources, meanwhile the importance and intensity of facilitation increases with increasing low air temperature stress. The patterns of competition intensity in our study adds the evidence that competition intensity does not remain unchanged or is not high in productive sites, as Tilman and Grime have predicted [1], [2], [11], [12]; but the pattern of facilitative intensity proves the theoretical prediction that facilitation becomes strong with increasing environmental severity [3]. In addition, we also found that the average percentage of species assembled by competition and facilitation both less than 30. This suggests that some ecological processes other than the positive or negative biotic interactions also simultaneously impact the species assemblage in these tropical cloud forest systems.
